# Relationship between microRNA-146a expression and plasma renalase levels in hemodialyzed patients

**DOI:** 10.1371/journal.pone.0179218

**Published:** 2017-06-14

**Authors:** Marcin Dziedzic, Tomasz Powrózek, Ewelina Orłowska, Wojciech Koch, Wirginia Kukula-Koch, Kinga Gaweł, Anna Bednarek-Skublewska, Teresa Małecka-Massalska, Janusz Milanowski, Beata Petkowicz, Janusz Solski

**Affiliations:** 1 Department of Laboratory Diagnostic, Medical University of Lublin, Lublin, Poland; 2 Department of Human Physiology, Medical University of Lublin, Lublin, Poland; 3 Department of Nephrology, Medical University of Lublin, Lublin, Poland; 4 Chair and Department of Bromatology, Medical University of Lublin, Lublin, Poland; 5 Chair and Department of Pharmacognosy with Medicinal Plants Unit, Medical University of Lublin, Lublin, Poland; 6 Department of Experimental and Clinical Pharmacology, Medical University of Lublin, Lublin, Poland; 7 Department of Pneumonology, Oncology and Allergology, Medical University of Lublin, Lublin, Poland; 8 Department of Oral Medicine, Medical University of Lublin, Lublin, Poland; Friedrich-Alexander-Universitat Erlangen-Nurnberg, GERMANY

## Abstract

**Background:**

microRNA (miRNA) belongs to the non-coding RNAs family responsible for the regulation of gene expression. Renalase is a protein composed of 342 amino acids, secreted by the kidneys and possibly plays an important role in the regulation of sympathetic tone and blood pressure. The aim of the present study was to investigate plasma renalase concentration, and explore the relationship between miRNA-146a-5p expression and plasma renalase levels in hemodialyzed patients.

**Methods:**

The study population comprised 55 subjects who succumbed to various cardiac events, 27 women and 28 men, aged 65–70 years. The total RNA including miRNA fraction was isolated using QiagenmiRNEasy Serum/Plasma kit according to the manufacturer’s protocol. The isolated miRNAs were analyzed using a quantitative polymerase chain reaction (qRT-PCR) technique. The plasma renalase levels were measured using a commercial ELISA kit.

**Results:**

In the group of patients with high levels of renalase, higher miRNA-146a expression was found, compared with those with low concentration of renalase. Patients with simultaneous low miRNA-146a expression and high level of renalase were confirmed to deliver a significantly longer survival time compared with other patients.

**Conclusions:**

miRNA-146a and plasma renalase levels were estimated as independent prognostic factors of hemodialyzed patients’ survival time. Patients with low miRNA-146a expression demonstrated a significantly longer survival time in contrast to the patients with a high expression level of miRNA-146a. Moreover, a significantly longer survival time was found in patients with high renalase activity compared with patients with low activity of the enzyme.

## Introduction

microRNA (miRNA) belongs to the non-coding RNAs family. Current estimates suggest that more than 60% of human protein-coding genes are regulated by miRNAs [1]. mRNA is not just a simple messenger between the DNA and various proteins, but is responsible for the regulation of genome organization and gene expression post-transcriptionally, as a single miRNA can bind and consequently regulate the expression of more than 100 different transcripts. miRNAs may be able to regulate up to 30% of the protein-coding genes in the entire human genome. miRNAs recognize their targets based on the sequence complementarity [2]. In humans, miRNAs mainly inhibit protein translation of their target genes and only infrequently cause a degradation or a cleavage of mRNA itself [2]. Previous studies denote that miRNA is crucial in regulation of practically all functions of a cell, from the initial proliferation, through the differentiation of the cell and up to its apoptosis [3]. The above conclusions are proven by further observations, shedding light on the occurrence of various diseases such as inflammatory and cardiovascular (CVD) malfunctions, or even cancers and the consequence of the functional abnormalities in the miRNA regulatory system [4]. Moreover, miRNAs are easily accessible for their concentration measurements in the plasma, serum, or also in urine due to their very specific expression profiles. The determination of these molecular biomarkers in the biological material may significantly improve the diagnosis of the patients and bring more data on the pathological mechanisms and also individually. miRNA is suggested to be one of the main factors of the regulation of gene expression, which has an impact on both physiological cardiac development and many pathological processes including cardiac arrhythmia, hypertension, heart failure, cardiac fibrosis, coronary artery disease, and myocardial infarction [3].

The chronic kidney disease (CKD) has been widely known as a risk factor for cardiovascular diseases. The CKD patients were often diagnosed with CVD, and died before being directed to dialysis [5]. However, 30% of the dialysis patients were suffering from CVD and as much as 50% died in hospitalization [6,7]. In addition, the CKD significantly affected the occurrence of diabetes and hypertension, which explains the high mortality rate among the dialysis patients. Cardiovascular risk cannot be completely elucidated by traditional risk factors. Several types of miRNAs regulate the functions of endothelial cells and peripheral signaling in the inflammatory processes, in particular miRNA-126 and miRNA-155. Although differentially expressed both are related to the occurrence of non-traditional risk factors of CKD [8]. Also, in their studies, Wang and co-investigators [8] have confirmed its ability to suppress the adhesion of leukocytes to the endothelial cells (ECs) and as a result to modify the inflammatory process. The role of miRNA-155 is based on the ability to regulate the adhesion molecules’ expression, which are present in the inflammatory ECs and in angiotensin α-mediated response to the inflammation [8]. According to previous research, three miRNAs (miRNA-126, miRNA-146, and miRNA-155) were described to play an important role in End-Stage Renal Disease (ESRD) patients for their ability to both induce the endothelial activation and increase the CVD risk [8]. Due to the demonstrated effects, the above-mentioned miRNAs have been considered as potent diagnostic markers.

Renalase is a protein made of 342 amino acids. Recently discovered as a new renal hormone, renalase-flavin adenine dinucleotide (FAD)–dependent amine oxidase [9] is secreted by the kidneys and can metabolize circulating catecholamines (CA), and possibly functions in the regulation of sympathetic tone and blood pressure. The renalase gene regulation mechanism, mostly the post-transcriptional one, has not been evaluated so far. The studies on the nature of these regulatory mechanisms are growing in significance over the recent years, and emphasizing the importance of the post-transcriptional miRNA genes regulation in this process. Based on the observations, various physiological dysfunctions, including the CVD, may be affected by the dysregulation of the non-coding small RNA fragments responsible for the gene expression [10,11,12]. The dysregulation of miRNAs functions evoked by the binding sites mutations may directly induce significant changes in the organism and lead to serious disease states. As an example, renalase was found to be directly related to the blood pressure and sugar level regulation and, when mutated, may lead to the occurrence of diabetes, strokes, or coronary heart disease [13,14,15]. The concept that renalase might be involved in the regulation of blood pressure is supported by the fact that the inactivation of the renalase (*RNLS*) gene in mice by homologous recombination is associated with elevated blood pressure and sympathetic activity in the absence of measurable changes in renal function [16]. The relationship between renalase and CA has been intensively studied since their discovery. Still we do not fully understand the possible impact of renalase on the occurrence of systemic diseases, such as cardiovascular dysfunctions, which often occur in hemodialysis (HD) patients. Therefore, there are many mechanisms underpinning the increased cardiovascular disorders. Recent studies have explored the relationship between variants in the *RNLS* gene and an increased risk of cardiovascular disorders [14]. *RNLS* gene resides on chromosome 10 (10q23.31). Stec et al. [17] investigated the association between renalase gene (rs10887800 and rs2576178) polymorphisms and risk of coronary artery disease (CAD) in HD patients. Authors [17] observed that renalase gene rs10887800polymorphism significantly increased the risk of CAD in HD. Moreover, the rs10887800 polymorphism affected the CAD risk independent of age, sex, and other CAD risk factors, including smoking, BMI, hyperlipidemia, arterial hypertension, and diabetes mellitus. In addition, Buraczynska et al. [13] demonstrated that renalase gene rs2296545 polymorphism is associated with hypertension in type 2 diabetes patients. Also, authors reported a strong association of the rs10887800 polymorphism with stroke in diabetic patients with hypertension and also in stroke patients without diabetes.

Our knowledge related to the cause of deaths in dialysis patients is rapidly expanding, still we do not fully understand the problem of high mortality in patients on dialysis. The major cause of death in HD patients is CVD, which constitutes 53% of causes of deaths in Poland [18]. In addition to traditional risk factors for CVD, such as hypertension and diabetes, lipid disorders are also important factors to consider. Also anemia, chronic systemic inflammation, accumulation of uremic toxins, disorders of calcium and phosphate, rapid changes in blood volume during HD, and volume overload of the circulatory system associated not only with renal failure (RF), but also with the presence of arteriovenous anastomosis are crucial. Most patients, who start their dialysis are hypertensive. Blood pressure (BP) control is an important target for reducing cardiovascular mortality [19]. Moreover, an elevated sympathetic activity is now recognized as an important mechanism involved in cardiovascular complications in humans [20]. Importantly, CVD is a major complication in patients with CKD and has a major impact on the morbidity and life expectancy of adults. Myocardial disease in CKD patients, as a part of a more generalized cardiovascular disorder, is manifested as left ventricular hypertrophy (LVH), diastolic dysfunction, and, to a lesser extent, systolic dysfunction [21].

Considering all these observations, the aim of the present study was to investigate renalase concentration and explore the associations between miRNA-146a expression and plasma renalase level in hemodialyzed patients.

## Materials and methods

### Study population

The study population comprised 55 subjects who succumbed to various cardiac events, 27 women and 28 men, aged 65 to 70 years. All patients underwent a clinical examination in the Department of Nephrology of the Medical University in Lublin, Poland. HD was performed on a selected group of patients 3 times a week for 3.5–4.5 hours. Low-flux dialyzers were applied in the studies. The bicarbonate dialysate contained a calcium solution at a concentration of 1.5 mmol/mL. The dialyzer blood flow rate ranged between 230 and 400 mL/min, while the dialysate flow rate was 500 mL/min. ESRD results were as follows: diabetic nephropathy (15 patients), glomerulonephritis (13 patients), hypertensive nephropathy (10 patients), connective tissue disease (6 patients), and polycystic kidney disease (4 patients). In the other 7 patients, the cause of death was not identified. In 34 patients, a concomitant ischemic heart disease was diagnosed, whereas heart failure was diagnosed in 21 patients; this group was qualified as New York Heart Association (NYHA) II (6 patients) and III (15 patients) functional class. Also, a few scores and parameters were determined for each patient, for example a comorbidity score (CS), which was described by the scale elaborated by Charlson et al. [22]. The HD adequacy was expressed by the Kt/V parameter [23], body mass index (BMI), normalized protein catabolic rate [24], and mean arterial pressure (MAP). The latter was determined based on the blood pressure measurement, recorded in a horizontal position, prior to HD. Well-controlled blood pressure was assessed according to the KDIGO guidelines as lower than 140/90 mmHg in HD patients before a hemodialysis session and lower than 130/80 mmHg after the session [6].

The study protocol was approved by the local Ethics Committee at the Medical University in Lublin, Poland (number: KE-0254/236/2015). All patients were informed about the aim of the study and a written informed consent was obtained from each patient qualified to participate in the study.

### miRNA isolation and miRNA quantification

Standard phlebotomy techniques were used to obtain the samples. All blood samples were collected into 5 mL EDTA-K_2_ covered tubes. The obtained plasma samples were collected in cry vial tubes and stored at –80°C until analyzed. The total RNA including miRNA fraction was isolated using Qiagen miRNEasy Serum/Plasma kit (Qiagen, USA) from 200 μl of plasma according to the manufacturer’s protocol. In the next step, the isolated miRNAs were analyzed using a quantitative polymerase chain reaction (qRT-PCR) technique. First, miRNAs were reverse transcribed to complementary DNA (cDNA) using the microRNA Reverse Transcription Kit (Applied Biosystems, USA) with miRNA primers, which provided specific and robust amplification only of the studied molecules. Reverse transcription reaction was conducted in TPersonal thermocycler (Biometra, Germany) in a total reaction volume of 15 μL according to the manufacturer’s protocol. Finally, cDNA of the studied miRNAs was amplified using TaqMan Universal Master Mix II with UNG (Applied Biosystems, USA) with TaqMan fluorescently labeled probes (Applied Biosystems, USA), targeting only studied miRNA-146a-5p in a total reaction volume of 20 μL in an Eco real-time PCR device (Illumina, USA), with the following reaction conditions: UNG activation—2 min at 50°C, polymerase activation—10 min at 95°C, and amplification—40 cycles: 15 s at 95°C and 1 min at 60°C. Ct values of examined samples were analyzed in Eco Study v4.0 (Illumina, USA) and then exported to Excel. All studied samples were normalized relative to U6 small-nuclear RNA (U6 snRNA), which was applied as an internal reaction control. The ΔCt and 2^-ΔCT^ analysis formula was used to assess expression of studied miRNAs in study set samples.

### Measurements of plasma renalase and IL-6 levels

The plasma renalase and IL-6 levels were measured using a commercial ELISA kit (USCN Life Science, Inc. Wuhan, China). For plasma renalase, the detection range was 3.12–200 ng/mL and the sensitivity was equal to the minimum detectable dose of this kit, i.e., <1.38 ng/mL. Furthermore, IL-6 levels detection range was 7.8–500 pg/mL and the sensitivity was equal to the minimum detectable dose of this kit, i.e., <3.2 pg/mL.

### Statistical analyzes

All statistical analyzes were conducted using Statistica 10.0 software (StatSoft, Poland) and MedCalc version 12.7 (MedCalc software, Belgium). All values were expressed as the mean and standard deviation (SD). The distribution of the analyzed variables was tested using the Shapiro—Wilk test. Fisher’s exact test was used to compare groups of patients with different miRNA expression and biochemical factors concentration. The Kaplan—Meier estimator with log-rank test analysis was used to correlate patients’ overall survival with different molecular and biochemical factors. Pearson’s correlation coefficient was applied to correlate miRNAs expression level with renalase concentration. Furthermore, the statistical relationship between the two variables was investigated using Spearman’s correlation coefficient R. In all tests, *P*-value < 0.05 was considered statistically significant for differences or correlations confirmation.

## Results

The main demographic and clinical characteristics of the patients included in the study are detailed in Table 1. From the conducted tests, the concentration of renalase was 81.91 ± 19.00 ng/mL. Patient’s gender was not found to affect significantly the plasma concentration of renalase as well as miRNA-146a (P > 0.05). In the group of patients with high levels of renalase, higher miRNA-146a expression was found, compared with those with low concentration of renalase. Moreover, the samples characterized by a low renalase level demonstrated lower miRNA-146a expression (P = 0.02). Longer life span was confirmed for those with high concentration of renalase compared with the patients with low plasma level of the enzyme (Median: 62 vs. 35 months; P = 0.01, HR = 1.897; 95%CI [1.063–3.383]) (Fig 1). Moreover, patients with low miRNA-146a expression level demonstrated a significantly longer survival time in contrast to the patients with high expression level of miRNA-146a (Median: 69 vs. 56 months; P = 0.430, HR = 1.728; 95%CI [0.995–3.002]) (Fig 2). Patients with simultaneous low miRNA-146a expression and high level of renalase were proven to deliver a significantly longer survival time compared with other patients (median: 77 vs. 39 months; P = 0.018, HR = 2.01; 95%CI [1.115–3.505]) (Fig 3). The IL-6 concentration has no effect on survival time (P = 0.507, HR = 1.323; 95% CI [0.546–3.210]). According to Pearson’s correlations analysis, the plasma levels of renalase were inversely related to miRNA-146a (R = –0.67; P = 0.03). Also, the Spearman rank correlation analysis revealed a significant negative correlation between the miRNA-146a concentration and the diastolic blood pressure (R = –0.3, P = 0.02) in the entire study group. However, the level of renalase did not correlate with blood pressure as well as MAP. Furthermore, according to Pearson’s correlations analysis, the plasma levels of IL-6 were slightly inversely related to miRNA-146a (R = –0.049; P = 0.02). Moreover, we observed that the expression level of miRNA-146a and IL-6 concentration had no significant effect on survival time (P = 0.694, HR = 1.215; 95%CI [0.412–2.971]).

**Fig 1:** Probability of overall survival change depending on renalase concentration level in hemodialyzed patients. High renalase concentration is a favorable prognostic factor of patients’ survival compared with patients with low concentrations of this enzyme (OS—62 vs. 32 months; p = 0.01; HR = 1.897).

**Fig 2:** Probability of overall survival change depending on miRNA-146a expression level in the studied group. Low miRNA-146a expression level is a favorable prognostic factor of patients’ survival compared with patients with high expression of this miRNA (OS—69 vs. 56 months; p = 0.430; HR = 1.728).

**Fig 3:** Probability of overall survival change depending on simultaneous analysis of renalase concentration and miRNA-146a expression level in hemodialyzed patients. Patients with simultaneous high concentration of renalase and low miRNA-146a expression demonstrate significantly higher OS compared with other studied patients (OS—77 vs. 39 months; p = 0.018; HR = 2.01).

**Table 1:** Baseline characteristics in long-term dialysis patients.

Parameter	Study group Mean ± SD n = 55	Males Mean ± SD n = 28	Females Mean ± SD n = 27
Age [years]	68.6±16.2	73.1±12.8	63.8±18.1
Time on HD [months]	49.44±34.3	53.48±37.15	46.12±32.53
BMI [kg/m^2^]	27.14±6.77	27.79±8.18	26.53±5.22
Kt/V	1.69±0.28	1.52±0.2*	1.84±0.27
Hemoglobin [g/dL]	10.4±1.3	10.6±1.0	10.26±1.53
EPO dose [U/kg]	66.9±37.3	62.4±38.6	71.0±36.5
CRP [μg/mL]	4.97±3.95	7.51±4.64*	3.4±2.56
IL-6 [pg/mL]	86.99±29.91	79.19±31.9	92.19±28.64
Total Calcium [mmol/L]	2.21±0.19	2.2±0.13	2.21±0.23
Phosphorus [mg/dL]	1.61±0.55	1.59±0.48	1.63±0.62
PTH [pg/mL]	632.9±510.3	478.9±208.5	738.8±627.0
Urea [mg/dL] Before HD	107.84±28.51	112.44±28.77	103.59±28.14
Urea [mg/dL] After HD	26.28±10.37	30.56±10.42*	22.33±8.78
Comorbidity score	6.96±3.19	7.57±3.22	6.47±3.18
Renalase [ng/mL]	81.91±19.0	83.46±16.26	80.49±21.45
miRNA-146a	0.86±0.19	0.88±0.18	0.84±0.2
Diastolic blood pressure [mm/Hg]	70.57±10.29	70.4±9.83	70.74±10.88
Systolic blood pressure [mm/Hg]	131.01±21.6	132.2±19.08	129.92±24.12
MAP [mmHg]	90.67±12.22	90.92±11.2	90.44±13.3

Data are presented as mean ± Standard Deviation (SD)

* P < 0.05—Compared males vs. females

BMI, Body Mass Index; Kt/V, number used to quantify hemodialysis treatment adequacy; EPO, erythropoietin; CRP, C-Reactive Protein; PTH, parathyroid hormone; HD, hemodialysis; MAP, mean arterial pressure.

## Discussion

One of the major challenges in hemodialysis patients is the identification of reliable biomarkers that can be measured routinely in easily accessible samples such as serum/plasma. The circulating miRNAs have been detected in both plasma/serum and other fluids of the body, which stayed in accordance with some recent studies, confirming their presence in extracellular fluids such as urine or blood in a stable form [25]. Two major transporting systems for miRNAs have been identified to date, which employ the exosomes and/or microvesicles, the apoptotic bodies, or possibly also other microparticles [26]. The miRNAs were also proven to be associated with lipoprotein complexes and non-vesicle associated proteins [27].

In a cross-study comparison, in HD patients of this study the plasma concentration of renalase was more markedly reduced than that (386.0±7.3 ng/mL) in the control group in a study by Zbroch et al. [28]. Moreover, the patients with low renalase level demonstrated a lower miRNA-146a expression. Based on the herein described results and the observations of Desir and Peixoto [29,30], decreased plasma levels of renalase may induce an elevated sympathetic tone in the studied ESRD patients. Moreover, a decreased concentration of the enzyme might lower the occurrence of cardiovascular complications and favorably result in a longer survival rate of patients [29]. Renalase degrades the circulating CA, causing a significant fall in blood pressure. However, in the present study, we did not observe any correlation between the level of renalase and blood pressure as well as of MAP. The obtained results were in agreement with Malyszko et al.’s study [31], which reported that renalase is secreted by the kidneys but it is also removed by dialysis to a much lesser extent. The same authors claimed that there is no clear relation between renalase and blood pressure, at least in patients with CKD and that it could not be confirmed that renalase was a monoamine oxidase or even an oxidase at all [32]. In contrast to the study of Beaupre et al. [33], who reported that renalase does not consume CA, renalase is not kinetically regulated by CA and is not isolated in an inhibited form, so it cannot be activated by blood plasma or CA. In addition, Beaupre and Brett et al. [33] suggested that blood has a very little concentration of the active renalase. This observation is consistent with its newly identified activity and suggests that renalase has an exclusively intracellular/metabolic role. Other authors also raised serious doubts regarding the putative catecholamine-degrading activity of renalase, suggesting that although renalase may have an important physiological role in the context of hypertension and cardiorenal disease, it appears unlikely for this enzyme to be mediated by a degradation of CA [34]. Wang et al. [35] showed that renalase promoted cell survival and showed a protective role against renal ischemia reperfusion injury in mice through the activation of intracellular signaling cascades, independent of its ability to degrade CA. More recently, Moran et al. [36] and Beaupre et al. [37] found that renalase does bind to adrenaline, but performs no catalytic transformation of it. Quelhas-Santos et al. [38] reported that renalase degrades CA, catalyzing the formation of aminochromes. Therefore, recombinant renalase exerts powerful and rapid hypotensive effects on rats through the improvement in circulating CA degradation. However, according to western blots and ELISA assays, incoherent results related to the blood renalase levels have been found, which triggers a further need to interpret the levels of this enzyme in patients suffering from kidney diseases more carefully [30]. Furthermore, the behavior of these antibodies and their epitopes in the western blots is not studied [30]. The tests may as well recognize other epitopes, which are normally not detectable by the polyclonal antibodies applied in the original studies [30,33,39,40]. As an example, ELISA may deliver false positive results, which are related to an increased concentration of renalase breakdown products in the advanced CKD patients or possibly a cross-reaction with other epitopes of the antibody [30]. Polyclonal antibodies in contrast to ELISA assay detect mainly the dimeric forms of the enzyme (~75 kDa) at a concentration of 4 μg/mL, and they preferably bind to the species of a higher molecular weight [30]. Considering the results of the recent studies, it might be concluded that the lower GFR values affect the accumulation and also formation of bigger multimers [30]. The two tests, ELISA and western blot assays, show coherent results in the patients with non-impaired renal functions. Based on these observations of Desir and Peixoto [30], a more careful analysis of the plasma renalase activities and levels in both healthy and diseased patients should be performed.

In this study, renalase was inversely related to miRNA-146a. Furthermore, in a group of patients with high levels of renalase, we found a higher miRNA-146a expression compared with the patients in whom low concentrations of renalase were found. A significantly longer survival time was found in patients with high concentrations of renalase compared with patients with low plasma levels of the enzyme. In addition, patients with low miRNA-146a expression demonstrated significantly longer survival time in contrast to patients with high expression level of miRNA-146a. Thus, our study showed that the expression of miRNA-146a was significantly reduced in all ESRD patients, which could influence the occurrence of significant clinical effects in patients [8]. However, the miRNA levels in the patients suffering from CKD could have decreased because of the kidney diseases occurring in the organism, which might have overpowered other pathological processes. Single miRNA measurements might not deliver satisfactory prediction. Multiple miRNAs regulated meaningful physiological functions of the organism [4]. These results support the hypothesis that the post-transcriptional regulation of the gene coding renalase, affected by miRNA-146a, undergoes interindividual variations on the cardiometabolic traits [41]. However, it is unknown whether circulating levels of miRNAs are affected in patients undergoing hemodialysis. miRNAs, which are circulating in the organism, are prone to influence the biosignaling functions, as they are coupled with protein transporters or with [42]. In this case, HD could have a meaningful impact on the miRNA levels in the organisms due to its ability to partially filtrate the proteins out of the blood stream, decrease the circulating levels of miRNAs in HD patients, and induce some biological effects. Emilian et al. [43] observed that circulating miRNA-499 levels were decreased after hemodialysis. Therefore, these observations mitigate the potential of miRNA-499 as a marker of myocardial injury in patients with ESRD. This study was limited by a small size of study group including the patients with ESRD. Thus, the authors could not investigate the association between miRNA levels and various grades of renal dysfunction. Evidence indicates that in pre-dialysis patients suffering from CKD, the circulating miRNAs levels are decreased, already suggesting an impaired miRNAs kinetics, possibly due to the dysfunctions of kidney filtration. These results are consistent with those of the study by Neal et al. [44], who showed that the levels of miRNA inversely correlated with a decrease of GFR and miRNA-155 levels, which were also related to the decreasing eGFR in patients with mild to severe CKD at their end stage renal disease receiving hemodialysis treatment. Also, the obtained results were in agreement with those found by Wang et al. [45], who saw a significant reduction in miRNA126 levels in ESRD patients. Moreover, Neal et al. [44] showed in their studies a visible degradation of the circulating RNAse, confirmed in the *ex vivo* exosomes study on the epithelium of colon cancer during its incubation with the plasma from CKD patients, in comparison with a control plasma [46]. The dialysis membranes should not allow any passage of larger molecules (30–40 kDa), although the HD process might have influenced the total quantity of the circulating miRNAs. In the works of Martino et al. [42], the effects of HD on the levels of circulating miRNA in blood were assessed after the collection of a spent dialysate. The authors confirmed that miRNA, as a very small particle, was not removed by the dialyzer membranes, also by those that were designed to filter out the middle-sized molecules. Besides, the authors [42] did not observe any impact of the HD procedure on the levels of circulating miRNA-21 and -210, compared with both pre- and post-dialyzer samples of blood. In conclusion, according to the authors, the HD therapy should not deplete the biologically active miRNAs from the patients’ circulation in acute kidney injury. However, it is a specific group of patients who delivered a whole series of metabolic disorders, which may have reflected the differences in the expression profile of circulating biomarkers, including those that are new miRNA.

Focusing on this inverse relation between renalase and miRNA-146a, the outcome of this study supports the hypothesis that renalase could play an important role in an increased cardiovascular risk. Our study showed that the patients with simultaneous low miRNA-146a expression and high level of renalase were characterized by a significantly longer survival time compared with other patients. In agreement with the data from the medical literature, miRNA-146 belongs to the miRNA family present in mammals, and also in humans. miRNA-146 has been proven to regulate and control the inflammation process, but also other processes, which involve the immune system [47]. miRNA-146 along with miRNA-155 was found to be an inflammation mediator. The expression of the former is induced by some inflammatory factors (IL-1,TNF-α) and it was confirmed to dysregulate a variety of targets, e.g., those involved in the pathways of a toll-like receptor, responsible for the cytokine system response [48]. miRNA-146 is operated in a ‘negative regulatory loop’ or in a feedback system that slightly controls the inflammatory responses [49]. The loss of functional miRNA-146 could have an impact on an individual to exhibit a chromosome 5q deletion syndrome [49]. However, the functions of miRNA-146 in proliferation and differentiation of Neural Stem Cells (NSCs) are poorly understood.

Thorough computational analyzes, which are often coupled with additional study validations, have confirmed that both miRNA-29 and miRNA-146 are important renalase expression regulators in both cultured kidney and neuronal cells [41]. The studies on the genetically modified hypertensive BPH mice showed the elevated levels of kidney miRNA-29b and the decreased levels of renalase, when compared with the hypotensive BPL species. These data indicated that miRNA-29b induced post-transcriptional regulation of renalase in this mouse model of human hypertension [41]. Also, the binding site of miRNA-146a is generated in the human *RNLS* 3′-UTR based on a widespread genetic variation (C/T; rs10749571), which was associated in a directionally concordant manner with a variety of several cardiometabolic phenotypes [41]. In view of these findings, the role of miRNAs in the regulation of the renalase genes was confirmed for the first time and showed the important causes of the molecular bases of cardiovascular and metabolic diseases [41]. Nonetheless, renalase is found to be secreted not only by the kidneys, but also by other tissues such as adipose tissue, cardiomyocytes, skeletal muscles, liver, the central nervous system, or the endothelium [50].

The circulating levels of miRNAs are affected in patients undergoing hemodialysis. The measurement of only the level of miRNA in HD patients will possibly not provide adequate information about the development of many pathological processes. HD patients are a specific group of patients who distinguished a whole series of metabolic disorders, which may have reflected the differences in the expression profile of circulating biomarkers, including miRNA. Consequently, a careful validation of HD implied changes should be done and reported in large clinical populations. The identification of miRNA represents the tip of a covered iceberg and the prediction of an individual miRNA. A deeper understanding of the involvement of miRNAs in HD patients is needed before these regulatory pathways can be explored as therapeutic approaches for CKD patients. miRNA expression is altered in various human disorders including systemic and metabolic diseases and especially neoplasms. To date, the most prominent issue is tissue-specificity of miRNAs. Because of the potency to regulate a wide range of targets by a single miRNA, it is hard to predict their function unequivocally. Therefore, the selection of miRNAs demonstrating tissue specificity. Studied miRNA-146a levels also meet the above limitations due to its involvement in the development of other diseases including cancer.

microRNA-146a is perceived as an inflammation marker in the age-related processes. It downregulates both the cellular senescence and also other inflammation inducing pathways [51]. Furthermore, microRNA-146a exhibits the above-described properties in the cells, which are engaged in vascular remodeling [52]. The obtained results showed that the IL-6 plasma concentration remained in an inverse relation with the miRNA-146a level. According to Kutty et al. [53], microRNAs such as miRNA-146b-5p and miRNA-146a are capable of inflammatory process regulation by the adulteration of cytokine signaling by the pathway of the nuclear factor-κB. Based on these observations, it can be stated that miRNAs are important markers of inflammatory diseases [54]. The influence on NF-κB, confirmed for both miRNA-146a and miRNA-146b-5p, has been explained by their ability to repress the translation of IRAK1 and TRAF6 [55]. According to Kutty et al. [53], IRAK1 was described as a target for both miRNAs in the RPE cell cultures. In addition, the studies of Bhaumik et al. [56] underline the negative influence of miRNA-146a/b on the secretion of IL-6 and IL-8, the mediators of inflammation, possibly suppressing the translation level with no relation to IRAK1 pathway, although there is a direct relation between the miRNA-146a/b upregulation and the immune system activity suppression through IRAK1 and TRAF6 mechanisms [57]. Both mediators as the components of IL-1 belong to the toll-like receptor signaling system, regulated (attenuated) by the NF-κB protein. Other mechanisms of action might be induced by the miRNA-146a/b to stimulate the production of cytokines. It could explain the lack of relations between the IL-6 level and the expression of miRNA-146a and lack of impact of the former on the survival time of studied patients.

The nature of this interaction needs to be elucidated by experimental and longitudinal clinical studies to recognize the possible presence of any cause—effect relationship between the miRNA levels and health condition.

## Conclusions

This experimental study on a group of patients targeted to explore the relation between the renalase activity and miRNA-146a expression. The investigation of miRNA plays a crucial role in the discovery of renalase activity through its post-transcriptional control of mRNA expression in hemodialyzed patients. Both miRNA-146a and renalase levels were estimated as independent prognostic factors of hemodialyzed patients’ survival time. Hemodialyzed patients with low miRNA-146a expression demonstrated a significantly longer survival time in contrast to the patients with a high expression level of this miRNA. Moreover, a significantly longer survival time was found in patients with high renalase activity compared with patients with low activity of the enzyme. Probably, an enhancement by simultaneously related inversion of studied markers resulted in a decreased possibility of early death in hemodialyzed patients. Therefore, dual assessment of both markers could enter a routine clinical implication with a higher diagnostic power of the experimental study group of patients. Further studies are needed on a larger group of patients to better elucidate the role of miRNA-146a with regard to renalase in hemodialyzed patients.
